The article "A Lightweight Semantic Segmentation Algorithm Based on Deep Convolutional Neural Networks" was retracted in 2023. Reasons: signs of a paper mill; suspected computer-generated content; unreliable results or conclusions; concerns about the data.

# A Lightweight Semantic Segmentation Algorithm Based on Deep Convolutional Neural Networks

**DOI:** 10.1155/2022/5339664

**Published:** 2022-09-06

**Authors:** Chengzhi Yang, Hongjun Guo

**Affiliations:** Laboratory of Intelligent Information Processing, Suzhou University, Suzhou 234000, Anhui, China

## Abstract

With the development of deep learning theory and the decrease of the cost of acquiring massive data, the image semantic segmentation algorithm based on Convolutional Neural Networks (CNNs) is gradually replacing the conventional segmentation algorithm by its high accuracy segmentation performance. By increasing the amount of training data and stacking more convolutional layers to form Deep Convolutional Neural Networks (DCNNs), a neural network model with higher segmentation accuracy can be obtained, but it faces the problems of serious memory consumption and long latency. For some special application scenarios, such as augmented reality and mobile interaction, real-time processing cannot be performed. To improve the speed of semantic segmentation while obtaining the most accurate segmentation results as possible, this paper proposes a semantic segmentation algorithm based on lightweight convolutional neural networks. Taking the computational complexity and segmentation accuracy into account, the algorithm starts from the perspective of extracting high-level semantic features and introduces a position-attention mechanism with richer contextual information to model the relationship between different pixels, avoiding the convolutional local perceptual field to be too small. To recover clearer target boundaries, a channel attention mechanism is introduced in the decoding part of the model to mine more useful feature channel information and effectively improve the fusion of low-level features with high-level features. By verifying the effectiveness of the above model on a publicly available dataset and comparing it with the more popular semantic segmentation methods, the model proposed in this paper has higher semantic segmentation accuracy and reflects certain advantages in objective evaluation.

## 1. Introduction

There are diverse targets in images, differences in sizes, and lighting conditions of the same object, and similar features among different objects, which increase the difficulty of semantic segmentation and are prone to confusion of organisms, so a broader range of feature information is needed to complete segmentation [1]. Convolutional neural networks have strong local perceptual abilities but are poor in acquiring global features. At the same time, the resolution of the feature map gradually decreases with the increasing number of network layers, and the extracted features change from figurative features such as texture and color to increasingly abstract feature information, so detail information is missing. The loss of detail information leads to coarser segmentation result, and there are also problems such as incomplete object contours [2].

In computer vision systems, image semantic segmentation is a difficult task. Among the deep learning methods, the techniques to implement the image semantic segmentation task are divided into two categories: one is the image semantic segmentation method based on region classification; the other is the image semantic segmentation method based on pixel classification. The region classification-based image semantic segmentation method is a method based on conventional methods combined with deep neural network structures. This method is to segment the input image into target candidate blocks according to certain rules, and then use deep neural networks to semantically classify the candidate blocks and label the classification to the original image [3]. Since the semantic segmentation methods based on region classification have problems such as blurred segmentation boundaries and slow running speed, thus prompting researchers to invest a lot of effort in pixel-level-based image semantic segmentation methods. The current pixel-level-based methods are divided into two modes: a fully supervised mode; and a semisupervised mode. The semantic segmentation method in fully supervised mode means that manually labeled tags are required as the input samples, and the label data of each pixel in the image is first read after input, and then the label data are used to train the deep neural networks, and the trained neural networks are used for semantic segmentation [4]. The main methods for semantic segmentation of images in fully supervised mode are currently based on fully convolutional neural networks, methods based on optimized convolutional structures, methods based on codecs, methods based on probabilistic graphical models, methods based on feature fusion, methods based on convolutional neural networks, and methods based on adversarial generative networks. Due to the increasing width and depth of network layers, convolutional neural networks are getting deeper and deeper; however, deep convolutional neural networks require a lot of manual intervention, and it is very time-consuming to collect labeled data sets manually, so semantic segmentation of images in semisupervised or weakly supervised mode has become popular at present [5]. The current mainstream semisupervised or weakly supervised image semantic segmentation methods are classified into image-level labeling, multilevel labeling, and bounding box labeling methods. DeepLab network is a novel deep neural semantic segmentation network proposed after the fully convolutional semantic segmentation network, which has good advantages over the previously proposed semantic segmentation networks; recently the concept of attention mechanism has been proposed in academia, aiming to use the attention mechanism to simulate human vision and thus to provide an intuitive interpretation of the network model [6]. In problems involving language or vision, some parts of the input will be more helpful for decision-making than others. The DeepLab v2 network introduces three new ideas in the model based on the shortcomings and deficiencies of the FCN network: Atrous Convolution (also known as Dilated Convolution), Atrous Spatial Pyramid Pooling, and Full-connected Conditional Random Field (CRF) [7].

This paper focuses on proposing a new parallel multibranching module for capturing contextual information to solve the problem of comparative dependence on square convolution and pooling operations, which lack the ability to perceive anisotropic contextual information. In order to better mine the channel information of the network output feature map, a channel attention module is introduced in the decoder of the network to ensure good performance and low computational complexity of the network.

## 2. Related Works

The success of AlexNet, VGG, GoogleNet, and ResNet's convolutional neural network for image classification and target detection has inspired researchers to explore the field of semantic segmentation with deep learning methods [8]. The key advantages of deep learning make it superior to conventional semantic segmentation methods. The pixel points of the images in the dataset are labeled one by one, and the results of semantic segmentation are obtained by end-to-end supervised training with CNNs, without the complicated processes of image processing, manual feature design, and feature extraction, so the successful semantic segmentation methods in recent years have been studied based on deep learning [9]. In recent years, the more successful semantic segmentation techniques are fully convolutional networks. This technique uses VGG as the network infrastructure and creatively replaces the fully connected layer at the end of the network with a fully convolutional layer, making the network directly output a segmentation result map with the same resolution as the original map. However, the segmentation map obtained by FCN is relatively coarse, so SegNet fills in the value of the maximum value and position of each pooling area before pooling by recording it and sets the value at that position and zero at other positions during up-sampling, but the obtained results are still not fine enough [10]. As the network structure deepens, the results of feature information extraction become more and more abstract, but at the same time, the obtained feature map resolution becomes smaller and smaller, and lacks a lot of spatial information. Most methods use direct recovery of the feature map to the resolution of the original map by bilinear interpolation, but the obtained results are mostly coarse. The convolutional operation of convolutional neural network extracts primary features such as texture and color in the shallow network and gets more abstract feature representation in the deep network, while the extracted information is based on local information features. The global information is necessary for segmentation, and the class to which the pixel belongs can be predicted more accurately by combining with the current environment [11, 12].

Compared with traditional image segmentation methods, the semantic segmentation algorithm based on CNN has great advantages in segmentation accuracy and visual performance. However, in some outdoor scenes, in the face of mutual occlusion of different objects, multiscale changes of the same target and weather changes, the task of image semantic segmentation still faces great challenges. Zhao et al. [13] developed an image semantic segmentation algorithm that combined fully convolutional network (FCN) with Simple Linear Iterative Clustering (SLIC). They also mixed the FCN semantic segmentation results with the superpixel information and introduced the superpixel semantic annotation. Zhang et al. [14] presented a novel semantic segmentation algorithm with DeepLab v3+ and superpixel segmentation algorithm-quick shift, which can further refine the semantic segmentation results. Meng and Choi [15] designed a semantic segmentation algorithm for point clouds based on the PointNet architecture. Their approach also applied the PointSIFT module, which can encode polydirectional information and adapt to the proportions of the shape being considered. Qiang et al. [16] proposed an object detection algorithm by jointing semantic segmentation (SSOD) for images. They constructed a feature extraction network that mixed the hourglass structure network with an attention mechanism layer to extract multiscale features and allowed the algorithm for multitask learning. Liu et al. [17] proposed an image semantic segmentation algorithm based on a deep neural network. Based on the Mask Scoring R-CNN, this algorithm used a symmetrical feature pyramid network and added a multiple-threshold architecture to improve the sample screening precision. Jiang and Li [18] proposed an improved semantic segmentation method for remote sensing images based on neural network. Based on residual network, it changed the dilated convolution kernels before extracting the correlations between geophysical objects, thus improving the segmentation accuracy and used a pixel-level method to achieve semantic segmentation. Girisha et al. [19] proposed an enhanced encoder–decoder based CNN architecture (UVid-Net) for unmanned aerial vehicle (UAV) video semantic segmentation. This advanced algorithm greatly enhanced the accuracy of the localization. Gharghabi et al. [20] presented a multidimensional algorithm, which was domain agnostic, had only one, easily determined parameter, and could handle data streaming at a high rate. Jiang et al. [21] designed Random-Walk-SegNet (RWSNet), a semantic segmentation network based on SegNet combined with random walk. It took SegNet as the basic architecture and adopted the sliding window strategy, realizing high-performance semantic segmentation of remote-sensing images. Yi et al. [22] trained the semantic segmentation neural network in different scenarios to obtain the models with the same number of scene categories, and experiments showed that the results of scene-aware semantic segmentation were much better than semantic segmentation without considering categories. Yang and Yu [23] introduced the progression of object detection and semantic segmentation in medical imaging study. They also discussed how to accurately define the location and boundary of diseases. Tan et al. [24] proposed a novel framework called joint 3D semantic-instance segmentation via multiscale semantic association and salient point clustering optimization, and designed a Multi-scale Semantic Association (MSA) module to explore the constructive effect of the context information for semantic segmentation. Jiang et al. [25] proposed a contouraware network for semantic segmentation via adaptive depth. They also constructed an adaptive deep model that could adaptively determine feedback from neural network and forward processes. Su and Wang [26] proposed a novel and practical convolutional neural network for effective semantic segmentation. It was comprised of three modules, namely broadening the residual convolutional neural network module, refining the residual feature pyramid module, and rolling the guidance edge retention layer module. Wu et al. [27] proposed a special semantic segmentation network by simulating the ventral and dorsal pathways of the brain visual cortex, which greatly enhanced the extraction of semantic information, and effectively improved the problem of spatial information loss during segmentation. Some classical image segmentation methods, such as FCN, SegNet, in order to pursue high segmentation accuracy, lead to complex models and high requirements for computing resources, which are not conducive to the use of semantic segmentation algorithms on resource constrained embedded devices. Because of its simplified model structure, lightweight semantic segmentation algorithm has the advantages of small amount of computation and fast segmentation speed, and can run in devices with limited computing resources. Therefore, the lightweight semantic segmentation method not only has practical application prospects but also promotes the improvement of segmentation algorithm.

## 3. Improvement of Image Semantic Segmentation Algorithm for DeepLabV3+

### 3.1. DeepLabV3+ Algorithm

The DeepLab algorithm is a model that focuses on semantic segmentation and introduces multiscale features, designs convolution and pooling operations with different parameters to obtain feature maps of different sizes, and efficiently fuses the obtained feature maps in the network model to improve the training performance of the whole network model. DeepLabV3+ algorithm is one of the more popular network model structures for the field of image semantic segmentation. The general construction of the DeepLabV3+ algorithm is shown in Figure 1 [28].

DeepLabV3+ is based on the structure of DeepLabV3, with a simple and efficient decoding module to refine the feature information and improve the segmentation effect. In the encoder part, the improved Xception model is used as the backbone network to extract different feature information in the image through the depth-separable convolution operation of different channels in the Xception model, and then the 1 ∗ 1 convolution and 3 parallel 3 ∗ 3 null convolutions with void rates of 6, 12 and 18, respectively, in the spatial pyramid pooling module and the global average pooling operation are used. After processing, and channel compression by 1 ∗ 1 convolution, the high-level semantic information is obtained. In the decoder part, the feature maps extracted from the input layer of the backbone network are first downscaled using 1 ∗ 1 convolution, after which they are fused with the high-level features obtained after encoder up-sampling, and then the spatial information in the feature maps is recovered using several 3 ∗ 3 convolutions and the target boundaries are refined using bilinear up-sampling to obtain the final segmentation result maps.

In the implementation of the DeepLabV3+ algorithm, the depth-separable convolution layer is proposed to replace the original maximum pooling layer, and the depth-separable convolution replaces the empty convolution operation in the Xception network model and decoder module, respectively, which can effectively by combining the ideas of depthwise conv and pointwise conv instead of null convolution, the computational complexity of the model in the training process can be effectively reduced to achieve a faster and stronger coder–decoder network.

### 3.2. Improvement of DeepLabV3+ Image Semantic Segmentation Algorithm

In order to improve the quality of feature map and solve the problems ignored in Deeplabv3+ algorithm, such as the different importance of features displayed in different feature maps, the loss of a large amount of detail information, and the impact on the final segmentation effect, this paper proposes an image semantic segmentation method based on improved Deeplabv3+. According to different levels of feature map and different attention mechanism modules, the image semantic segmentation algorithm adopts encoding–decoding structure, the backbone network still adopts Xception model. The attention mechanism module is divided into channel attention (CA) module and spatial attention (SA) module. Channel attention is added to the encoder and spatial attention is added to the decoder.

The input image is first extracted by the depth-separable convolutional layer of different channels in the Xception model; second, the feature map obtained from the output layer is processed in parallel by the atrous spatial pyramid pooling module and the channel attention module, and the specific implementation process is as follows: (1) the 1 × 1 convolution, the 3 × 3 null convolution with 3 null rates of 6, 12 and 18, respectively, and the global average pooling are used in the atrous spatial pyramid pooling module. After processing, stitching and fusion are performed, and then 1 pair of convolution is used for dimensionality reduction. (2) The feature map obtained through the network model is first reduced to 256 by 1 × 1 convolution, and then the channel attention module is used for weighting; finally, the feature map processed by ca and the feature map reduced by atrous spatial pyramid pooling module are summed for feature fusion to extract the rich contextual information to obtain effective high-level features.

Because the encoder part obtains high-level features through the parallel way of channel attention module and spatial pyramid pooling module, in order to obtain more efficient segmentation effect, this paper adopts the way of connecting channel attention module and spatial pyramid pooling module in series. In the encoder, the input image goes through the depth-separable convolution layer of different channels in the Xception model for feature extraction, and the feature map output from the output layer is processed by the atrous spatial pyramid pooling module and the channel attention module. Firstly, using the 1 × 1 convolution in the atrous spatial pyramid pooling module, the void rate of 6, 12, and 18, respectively, and global average pooling operation, respectively, and then perform feature fusion operation on them, and reduce the number of feature map channels from 2048 to 256 by 1 × 1 convolution of the obtained feature map again, and second, fuse the feature map obtained in atrous spatial pyramid pooling module using the channel attention module and perform weighting operation on them to obtain effective high-level features.

### 3.3. DeepLab Network Model Based on Attention Mechanism Module

The formula according to the SE attention module is

(1) $$\begin{array}{c} f_{\left\{w_{1},w_{2}\right\}}\left(y\right)=W_{2}\text{Relu}\left(W_{1}y\right), \end{array}$$

*W*_1_ and *W*_2_ are the fully connected parameter matrices, *y* is the output weight of the feature map after global average pooling, Relu is the activation function. The use of fully connected layers *W*_1_ and *W*_2_ reduces the complexity of the model and consequently the dimensionality; this indirect approach also destroys the direct correspondence between channels and weights.

This paper proposes the module which aims to ensure the multidimensional relationship between channels and weights as well as not to increase the complexity of the whole module computation. The formula for the module is the following:

(2) $$\begin{array}{c} \omega =\sigma \left(Wy\right), \end{array}$$

*y* is still the output weight after global average pooling, *σ*(*•*) is the activation function. *W* is the vector matrix used to calculate the channel attention. Its form is

(3) $$\begin{array}{c} \left[\begin{array}{c} W^{1,1}\\ \begin{array}{c} \cdots \\ \cdots \\ 0 \end{array} \end{array}\begin{array}{c} \cdots \\ \begin{array}{c} W^{2,2}\\ \cdots \\ \cdots \end{array} \end{array}\begin{array}{c} W^{1,k}\\ \begin{array}{c} 0\\ \cdots \\ 0 \end{array} \end{array}\begin{array}{c} 0\\ \begin{array}{c} W^{2,k+1}\\ \cdots \\ 0 \end{array} \end{array}\begin{array}{c} 0\\ \begin{array}{c} 0\\ \cdots \\ \cdots \end{array} \end{array}\begin{array}{c} \cdots \\ \begin{array}{c} \cdots \\ \cdots \\ W^{C,C-K+1} \end{array} \end{array}\begin{array}{c} \cdots \\ \begin{array}{c} \cdots \\ \cdots \\ \cdots \end{array} \end{array}\begin{array}{c} 0\\ \begin{array}{c} 0\\ \cdots \\ W^{C,C} \end{array} \end{array}\right]. \end{array}$$

The matrix *W* involves *K* × *C* parameters, and the matrix avoids the complete independence of the different group categories in the SE module. For the weight *y*, in order to simplify the calculation and avoid dimensionality reduction, only the information interaction between it and its *k* neighboring elements is considered here and calculated as follows:

(4) $$\begin{array}{c} \omega_{i}=\sigma \left(\overset{k}{\underset{j=1}{\sum }}w_{i}^{j}y_{i}^{j}\right),y_{i}^{j}\in \Omega_{i}^{k}. \end{array}$$

To further improve performance, let all channels share weight information, that is,

(5) $$\begin{array}{c} \omega_{i}=\sigma \left(\overset{k}{\underset{j=1}{\sum }}w^{j}y_{i}^{j}\right),y_{i}^{j}\in \Omega_{i}^{k}. \end{array}$$

Therefore, if all channels share the weight information, then the information sharing and interaction between channels can be achieved by one-dimensional convolution with a convolution kernel of size *k*:

(6) $$\begin{array}{c} \omega_{i}=\sigma \left({\text{Convld}}_{k}\left(y\right)\right), \end{array}$$

Convld means the one-dimensional convolution operation, which involves only *k* parameter information, and when *k*=3, the module can achieve the same effect as the SE module but with a lower model complexity. This approach of capturing cross-channel information interactions without downscaling ensures performance results and low complexity of the module.

Since the module aims to properly capture the local cross-channel information interaction sharing, it is necessary to determine the approximate region *k* (the size of the convolutional kernel in a 1D convolution) of the channel interaction. Although manual optimization can be performed for different convolutional blocks with different number of channels in different convolutional neural network architectures to achieve the optimal solution for information interaction, cross-validation tuning can be resource-intensive if performed manually and manually. Grouped convolution methods are known to have been successfully used to improve deep convolutional network architectures: for a fixed number of groups, high-dimensional (low-dimensional) channels are proportional to long-distance (short-distance) convolutions. Similarly, it follows that the coverage *k* of cross-channel information interactions should also be proportional to the number of channel dimensions *C*. That is, there may be a mapping relationship *φ* between region *C* and channel *C*:

(7) $$\begin{array}{c} C=\varphi \left(k\right). \end{array}$$

The simplest mapping method is the linear mapping relationship. Due to the limitations of linear functions in deep neural networks for some features and the fact that the channel depth is generally an exponential multiple of 2, an exponent with a base of 2 is used to represent the nonlinear mapping relationship:

(8) $$\begin{array}{c} C=\varphi \left(k\right)=2^{\left(\gamma \times k-b\right)}. \end{array}$$

In this way, given the channel dimension  *C*, the one-dimensional convolutional kernel size k can be derived from the following equation:

(9) $$\begin{array}{c} k=\psi \left(C\right)={\left|\frac{{\text{log}}_{2}\left(C\right)}{\gamma }+\frac{b}{\gamma }\right|}_{\text{odd}}, \end{array}$$

|*t*|_odd_ is the nearest odd number to *t*. *γ* and *b* are hyperparameters that need to be set, which are related to the structure of the network being joined. In the DeepLab network to be optimized, it is set to *γ*=2, *b*=1.

At the same time, since the module only introduces a one-dimensional convolutional kernel size *k* as a parameter, it does not introduce a large number of parameters when the attention mechanism module is introduced into the network, and only one one-dimensional convolutional computation and dimensional expansion operations are calculated in terms of computation.

After performing a null convolution, after global average pooling (GAP) without dimensionality reduction, a one-dimensional convolution of convolution kernel size is used to extract cross-channel interaction information of neighboring elements between channels, where the *k*-value indicates the coverage of local cross-channel interactions, that is, how many neighboring elements are involved in the attention prediction of that channel. The tensor of the one-dimensional convolution output is passed through the activation function *q*, which has different weight shares of the attention prediction attributes; the tensor is matrixed with the original null convolution channel to obtain an output with the same dimensions as the original input and with channel attention prediction. It is proved that this method ensures the learning efficiency and computational results of the model.

In order to compare the effect before and after the improvement, the DeepLab network model based on the module is constructed in this paper. In order to avoid the easy overfitting problem caused by the unavailability of the pretrained network model after the module is added to the backbone network, the module is added to the structure of the decoder part of the DeepLab network, and this is embedded in the feature pyramid after the convolution of the voids, and then multiscale feature fusion is performed after the attention mechanism prediction, as shown in Figure 2. In addition to using different backbone networks VGG-16 network and Res-50 network in the experiments with and without the addition of module, the Res-101 network with deeper structure is also added. Since these three networks have more layers, in order to achieve better classification results on the SBD and ADE20K datasets, the input image size was preset to 321 × 321 when conducting the computer simulation experiments, and then the images were fed into the network for learning training and validating the predictions.

In this paper, the proposed algorithm combines the advantages of depth-separable convolution with the attention mechanism and uses different attention modules to effectively fuse the low-level and high-level features for different levels of important features in the input image. In the process of implementation, all the empty convolution operations in the attention mechanism are replaced by the deep separable convolution operations, and as the number of features to be extracted gradually increases, the deep separable convolution can save more parameters and improve the computational speed of the training model compared with the empty convolution.

## 4. Experimental Results and Analysis

### 4.1. Data Sources and Evaluation Indicators

#### 4.1.1. Data Sources

The SBD dataset is an enhanced version of the VOC 2011 dataset, which contains the annotation of 11355 images from the Pascal VOC 2011 data set. The 11355 images in the SBD are completely selected from the pictures in the VOC 2011 dataset, and more of them are annotated. The category is also the same as VOC 2011 (21 categories). ADE20k is composed of 27000 images from the sun and places data sets. ADE20k consists of more than 3000 object categories, many of which comprise the categories of parts and components of objects, as well as the categories of parts and components of parts and components, such as auto parts, door parts, and windows. The ID of the instance is also marked in ADE20k, which can be used for instance segmentation.

#### 4.1.2. Evaluation Indicators

In this paper, we use mean Intersection over Union (mIoU) to evaluate the network performance, which is a standard measure of semantic segmentation accuracy. mIoU is larger, which means better segmentation. In semantic segmentation, the two sets in IoU represent the predicted segmentation and the true value (GT) of the segmentation. The IoU of each category is calculated first, which is the intersection of the two sets of the predicted and true values of the model segmentation and the overlap ratio of its concurrent set, and then averaged to obtain mIoU. The expression is shown as

(10) $$\begin{array}{c} \text{mIoU}=\frac{1}{k+1}\overset{k}{\underset{t=0}{\sum }}\frac{TP}{TP+FP+FN}. \end{array}$$

TP denotes positive samples predicted to be positive, FN denotes positive samples predicted to be negative, FP denotes negative samples predicted to be positive, and TN denotes negative samples predicted to be negative.

### 4.2. Model Parameter Tuning

Before starting to train the model, the weights of the network are initialized, and the weights of the remaining convolutional layers of the network to be learned are initialized to obey a Gaussian distribution with mean 0 and standard deviation 0.01, and the bias is set to 0. During the training process, the weights are updated iteratively according to the chain rule, and this fine-tuning scheme greatly reduces the convergence time during the training of the semantic segmentation model.

In the process of model design, the ReLU function is used in the activation layer and the Softmax function is used in the loss layer. During the training of the semantic segmentation model, the input is the predicted value of the network with the real label map. To prevent overfitting, the weight decay rate decay = 0.0001. The function is the cross-entropy loss function:

(11) $$\begin{array}{c} \text{loss}=-\overset{N}{\underset{\text{t}}{\sum }}{\text{y}}_{\text{i}}\log\left(\frac{{\text{e}}^{{\text{z}}_{\text{i}}}}{{\sum^{}}_{\text{j}=1}^{\text{n}}{\text{e}}^{{\text{z}}_{\text{j}}}}\right). \end{array}$$

The optimizer uses the Stochastic Gradient Descent (SGD) and Momentum method (Momentum = 0.9) with the following equation for the optimization function:

(12) $$\begin{array}{c} w_{t}=w_{t-1}+\text{momentum}\times v-lr\times \Delta w. \end{array}$$

In (12), lr denotes the learning rate, Δ*w* denotes the first-order derivative of the loss function with respect to the weights, denotes the update rate, and *w*_*t*−1_ and *w*_*t*_ denote the weights of the previous iteration and the updated weights values, respectively. In the process of gradient update, the momentum term can be increased for dimensions with the same direction out at the gradient point, while the momentum term is reduced for dimensions that change direction at the gradient point. Therefore, the optimization method of SGD and momentum helps to reduce the training time.

In the later stages of training, the decay of the learning rate lr contributes to the stability of convergence, and the learning strategy in this paper is as follows:

(13) $$\begin{array}{c} lr={\text{base}}_{lr}\times {\left(1-\frac{\text{iter}}{\text{maxiter}}\right)}^{\text{power}}. \end{array}$$

In (13), power is 0.95, base_lr is 0.007, maximum iterations is 40 k, set the output step to 15, and batch size to 10. The following shows the training results with different parameter settings. Figures 3(a) and 3(b) show the loss curve (Loss) and accuracy curve (mIoU) obtained from the model training under different experimental schemes, respectively, on SBD dataset.

From Figure 3 we can see that the model converges basically after 30 k iterations, and the loss value converges to a smaller value when the initial learning rate base_lr is 0.007; the initial learning rate is set too small at the beginning, which leads to the slow convergence of SGD + momentum method, and the final accuracy is poor.

### 4.3. Comparative Experimental Results and Analysis

Under the experimental conditions, semantic segmentation models of different backbone networks, including FCN-8s, DeepLabV3, and DeepLabV3+, were trained under the same configuration using the same data enhancement (flipping and multiscale), and the methods in this paper were compared with these semantic segmentation methods.  Table 1 shows the results of the comparison experiments on the SBD dataset.

As seen from Table 1, the method in this paper takes good care of the number of parameters, computation and performance of the network, and achieves a good balance between segmentation accuracy and efficiency. In terms of segmentation accuracy, this method has different degrees of advantages over FCN-8s (VGG16), DeepLabV3 (MobileNetV1), and DeepLabV3+ (ResNet50) in Table 1.

When training this paper's model on the ADE20k dataset, the images were cropped to 768 × 768, the batch size is 10 and the maximum iterations is 30 k for the maximum number of iterations, and the rest of the hyperparameters were set as above. The loss (Loss) curve as well as the accuracy curve (mIoU) plots during model training is shown in Figure 4. The final mIoU of the method in this paper on the ADE20k is up to 72.8%.

## 5. Conclusion and Future Work

In this paper, we study the backbone network, atrous spatial pyramid pooling module and decoder in DeepLabV3+, analyze the limitations of each part, introduce the channel attention module, and propose an image semantic segmentation algorithm based on spatial attention mechanism to address the problem of insufficient segmentation accuracy of existing algorithms. The proposed algorithm uses channel attention to weight the feature maps obtained from the backbone network, and then fuses them with the feature maps processed by the atrous spatial pyramid pooling module to obtain rich contextual information and get high-level features; spatial attention is used to fuse the two low-level features with the high-level features processed by convolution, respectively, to filter a large amount of background information and highlight feature points. In addition, the feature map is linearly transformed using the feature transformation principle to reduce unnecessary convolution operations. In addition, the shallow feature map information is reused in the decoder section using a shortcut connection to enrich the image details. The experimental results verify the effectiveness of the proposed algorithm in this paper, which has obvious advantages in terms of computational complexity and segmentation accuracy compared with similar algorithms.

The efficient semantic segmentation method based on DCNN is also based on the convolutional and pooling layers of CNN, and the network architecture is optimized. However, the activation layer is also an important part of the deep network design. Therefore, the impact of the activation function on the model performance will be further investigated in the subsequent study. Since the great success of transformer in natural language processing tasks has been explored in the field of computer vision, using transformer for semantic segmentation vision tasks to reduce the complexity of the structure and explore scalability and training efficiency will also be a direction for future research.

## Figures and Tables

**Figure 1:** DeepLabV3+ algorithm structure diagram.

**Figure 2:** DeepLab network decoder model based on channel attention module.

**Figure 3:** Training of the model proposed in this paper on the SBD dataset: (a) loss curve and (b) accuracy curve.

**Figure 4:** Training of the model proposed in this paper on the ADE20k dataset (a) loss curve (b) accuracy curve.

**Table 1:** Comparison results of each model on the SBD dataset.

Segmentation method	Backbone network	mIoU (%)
FCN-8s	VGG16	63.72
DeepLabV3	MobileNetV1	73.56
DeepLabV3+	ResNet50	76.18
This model	MobileNetV2	79.03

## Data Availability

The data supporting the findings of this study are included within the article.
